This article has been retracted.

# 27-Hydroxycholesterol increases α-synuclein protein levels through proteasomal inhibition in human dopaminergic neurons

**DOI:** 10.1186/s12868-018-0420-5

**Published:** 2018-04-03

**Authors:** Jared Schommer, Gurdeep Marwarha, Trevor Schommer, Travis Flick, Jonah Lund, Othman Ghribi

**Affiliations:** Department of Biomedical Sciences, School of Medicine and Health Sciences, University of North Dakota, 1301 N Columbia Rd Stop 9037, Grand Forks, ND 58202 USA

**Keywords:** 27-Hydroxycholesterol, Αlpha-synuclein, Liver X receptor, Parkinson’s disease, Dopaminergic neurons, Proteasomal dysfunction

## Abstract

**Background:**

Accumulation of the α-synuclein (α-syn) protein is a hallmark of a group of brain disorders collectively known as synucleinopathies. The mechanisms responsible for α-syn accumulation are not well understood. Several studies suggest a link between synucleinopathies and the cholesterol metabolite 27-hydroxycholesterol (27-OHC). 27-OHC is the major cholesterol metabolite in the blood that crosses the blood brain barrier, and its levels can increase following hypercholesterolemia, aging, and oxidative stress, which are all factors for increased synucleinopathy risk. In this study, we determined the extent to which 27-OHC regulates α-syn levels in human dopaminergic neurons, the cell type in which α-syn accumulates in PD, a major synucleinopathy disorder.

**Results:**

Our results show that 27-OHC significantly increases the protein levels, not the mRNA expression of α-syn. The effects of 27-OHC appear to be independent of an action through liver X receptors (LXR), its cognate receptors, as the LXR agonist, GW3965, or the LXR antagonist ECHS did not affect α-syn protein or mRNA levels. Furthermore, our data strongly suggest that the 27-OHC-induced increase in α-syn protein levels emanates from inhibition of the proteasomal degradation of this protein and a decrease in the heat shock protein 70 (HSP70).

**Conclusions:**

Identifying 27-OHC as a factor that can increase α-syn levels and the inhibition of the proteasomal function and reduction in HSP70 levels as potential cellular mechanisms involved in regulation of α-syn. This may help in targeting the correct degradation of α-syn as a potential avenue to preclude α-syn accumulation.

## Background

Synucleinopathies are pathologically characterized by the abnormal accumulation of α-syn protein in intracellular inclusions known as Lewy bodies. The role of α-syn in the pathogenesis of synucleinopathies is not well understood but extensive experimental data points to a neurotoxic role of high levels of the protein in its soluble and aggregated forms [1–4]. For the last decade, hyperlipidemia has been under scrutiny as a risk factor for synucleinopathy of Parkinson’s disease (PD) type [5–7]. However, while various studies showed an increased risk [8–10], other studies reported a decreased risk [11–13], or no association with high cholesterol levels [14, 15]. It may be possible that the conflicting results are indicative of the disturbances in the cholesterol oxidation derivative 27-OHC, not cholesterol per se, as the risk factor for PD. In addition to being a cholesterol oxidation product (oxysterol), 27-OHC is an active product that has a variety of biological functions. One of its main functions is to bind to liver X receptors (LXRs), thus affecting genes and proteins that are regulated by these receptors [16, 17]. LXRs, by means of gene transcription, regulate several metabolic pathways including lipid metabolism, glucose homeostasis, and inflammation [16]. LXRs regulate gene transcription by binding to promotors of genes and recruiting co-activators or co-repressors to enhance or repress the expression of target genes [16]. In support of our speculation of a link between synucleinopathies and 27-OHC are studies showing increased levels of a variety of cholesterol oxidation products (oxysterols), including 27-OHC, within the brains of patients with synucleinopathies [8, 18–22]. Oxysterol levels have also been shown to be increased in the circulation of hypercholesterolemic individuals [23, 24], with aging [5, 25], and with oxidative stress [26], all of which are risk factors for PD. Another interesting observation in support of a role of 27-OHC in brain neurodegeneration is that 27-OHC can cross the blood brain barrier while cholesterol cannot [19, 20, 27, 28]. This data points to a potential association between accumulation of the oxysterol 27-OHC and synucleinopathies. However, the potential mechanisms by which 27-OHC may affect α-syn levels and increase the risk for synucleinopathies remains to be determined. Ours [21, 22] and others [29] published data showed that 27-OHC increases the transcription of α-syn through activation of LXRs in human neuroblastoma SHSY-5Y cells. However, whether 27-OHC can also affect α-syn transcription in human dopaminergic neurons is yet to be demonstrated. Furthermore, whether the accumulation of α-syn involves the inhibition of its degradation by 27-OHC is not known.

α-syn has been shown to be degraded by the proteasome [30–32], and proteasomal dysfunction has often been implicated in PD [33, 34]. Currently, the extent to which 27-OHC inhibits the Ubiquitin-Proteasomal System (UPS) to increase α-syn accumulation remains to be shown. Heat shock proteins (HSPs) are one of the most structurally and functionally conserved proteins in evolution. In addition to their role in cellular stress, they are involved in the disassembly of protein aggregates and targeting of proteins for degradation. Increasing HSP70 has been shown to inhibit α-syn accumulation in PC12 cells [35]. In this study we aimed to investigate the effects of 27-OHC on both UPS and HSP70 protein levels. We found that 27-OHC increases α-syn protein levels independently of LXR, through proteasomal inhibition and HSP70 reduction in normal human dopaminergic neurons.

## Methods

### Materials

27-OHC (Cat. # 3907), the LXR agonist GW3965 (Cat. # G6295), and the proteasome inhibitor MG132 (Cat. # 1748) were purchased from Tocris (Minneapolis, MN, USA). The LXR antagonist Cholestan-5α, 6α-EPOXY-3β-OL sulfate sodium salt (ECHS, Cat. # C4136-000) was purchased from Steraloids Inc. (Newport, RI, USA). All cell culture reagents, with the exception of fetal bovine serum (Cat. # S11150H, Atlanta Biologicals, Lawrenceville, GA, USA), dibutyryl cAMP (Cat. # sc-201567 Santa-Cruz Biotechnology, Inc. Dallas, TX, USA), antibiotic/antimycotic mix (Cat. # 15240-062, Sigma Aldrich) and Poly l-Lysine (Cat. # P4707, Sigma Aldrich) were purchased from Applied Biological Materials (Richmond, BC, Canada). Human primary Dopaminergic Neuronal Precursor cells (Cat. # T4034), PriGrow IV medium (Cat. # TM004), Fibroblast Growth Factor 2 (Cat. # Z101455), Glial-Derived Neurotrophic Factor (Cat. # Z101055), and Epidermal Growth Factor (Cat. #Z100135) were purchased from Applied Biological Materials (Richmond, BC, Canada).

### Cell culture and treatments

Human primary Dopaminergic neuronal precursor cells were grown in PriGrow IV medium containing 5% fetal bovine serum, 10 ng/mL Fibroblast Growth Factor 2, 10 ng/mL Glial-Derived Neurotrophic Factor, and 1% Penicillin–Streptomycin. Cells were maintained at 37 °C in a saturated humidity atmosphere containing 95% air and 5% CO_2_. Cells were cultured and passaged for thirty days prior to differentiation. Plates were coated with Poly l-Lysine and the cells were plated at a density of 10^4^ cells per cm^2^ with differentiation media consisting of PriGrow IV, 5% fetal bovine serum, 10 ng/mL fibroblast growth factor 2, 10 ng/mL epidermal growth factor, and 100 µM dibutyryl cAMP for twenty-five days to allow for differentiation. Following differentiation, cells were incubated with ethanol vehicle (control), 0.5 µM 27-OHC (physiological concentration), and 1 or 10 µM 27-OHC (high concentrations) for twenty-four hours for the 27-OHC alone experiments. For experiments involving LXR agonist and antagonist cells were incubated with ethanol and DMSO vehicle (control), 10 µM 27-OHC, 10 µM GW3965, 10 µM ECHS, 10 µM 27-OHC + 10 µM ECHS for twenty-four hours. The concentrations we used are based on our previously published data in SHSY-5Y cells [21]. For experiments involving the proteasomal inhibitor MG132 cells were incubated with ethanol vehicle (control), 10 µM 27-OHC, and 1 µM MG132 for twenty-four hours. The half-life of α-synuclein has been estimated by pulse-chase experiments to be 26.5 h [36]. We chose MG132 for 24 h for this reason and because others have inhibited the proteasome for 24 h with MG132 prior to experimentation involving α-syn [36]. In all above mentioned treatments, three biological replicates were assigned to plates and were all utilized in the subsequent experiments including technical replicates. Cells were authenticated by Applied Biological Materials and tested negative for Mycoplasma contamination.

### LDH assay

The effect of 27-OHC, GW3965, ECHS, and 27-OHC + ECHS on cell toxicity was quantitatively determined by the measurement of lactate dehydrogenase (LDH) released from the cells into the medium 24 h post treatments using an LDH Assay (Promega, Madison, WI, USA) according to the manufacturer’s recommendations. Data were analyzed by comparison of the intensity of the absorbance in vehicle-treated cells to the treatments and subjected to one-way ANOVA. Data are expressed as individual values with mean ± SEM (n = 3 wells per one sample from three separate samples).

### Western blotting

Cultured human dopaminergic neurons were treated for 24 h with ethanol vehicle control, 0.5, 1, 10 µM 27-OHC in the initial experiments. In the second set of experiments cultured human dopaminergic neurons were treated for 24 h with ethanol and DMSO vehicle (control), 10 µM 27-OHC, 10 µM GW3965, 10 µM ECHS, 10 µM 27-OHC + 10 µM ECHS. For experiments involving the proteasomal inhibitor MG132 cells were incubated with ethanol vehicle (control), 10 µM 27-OHC, and 1 µM MG132 for twenty-four hours. Treated cells were washed with phosphate-buffered saline (PBS), followed by protein extraction with RIPA buffer. Protein concentrations were determined with the BCA protein assay reagent by standard protocol. Proteins (10 µg) were separated on sodium dodecyl sulfate–polyacrylamide gel electrophoresis gels, transferred to a polyvinylidene difluoride membrane (Bio-Rad, Hercules, CA, USA), and incubated overnight at 4 °C with the following antibodies: anti-α-synuclein rabbit antibody (Cat. # 2642S, RRID: AB_10695412) (1:500; Cell Signaling Danvers, MA, USA), anti-ATP-binding cassette transporter (ABCA1) (Cat. # Mo13101, RRID: AB_2220136) (1:500; Neuromics Minneapolis, MN USA), anti-HSP70 antibody (Cat. # PA5-28003, RRID: AB_2545479) (1:1000; Thermo Fisher Scientific Waltham, MA USA), and anti-Dopamine Transporter (Cat. #MAB369, RRID: AB_2190413) (1:1000; EMD Millipore Temecula, CA USA). Antibodies have been extensively validated by the companies of origin. β-Actin was used as a gel loading control. The blots were developed with Clarity Western ECL Substrate (Biorad, Hercules, CA). Bands were visualized on a polyvinylidene difluoride membrane on an Aplegen Omega Lum G System (Pleasanton, CA, USA) and analyzed by ImageJ (NIH, USA). The results were quantified by densitometry and represented as total integrated densitometric values. Data are expressed as individual values with mean ± SEM and includes determinations made in two separate experiments containing (n = 3) and technical replicates for all proteins except DAT which was one experiment (n = 2).

### Immunofluorescence

Human primary Dopaminergic neuronal precursor cells were grown in PriGrow IV medium containing 5% fetal bovine serum, 10 ng/mL Fibroblast Growth Factor 2, 10 ng/mL Glial-Derived Neurotrophic Factor, and 1% Penicillin–Streptomycin. Cells were maintained at 37 °C in a saturated humidity atmosphere containing 95% air and 5% CO_2_. Cells were cultured and passaged for thirty days prior to differentiation. Coverslips were coated with Poly l-Lysine and the cells were plated at a density of 10^4^ cells per cm^2^ with differentiation media consisting of PriGrow IV, 5% fetal bovine serum, 10 ng/mL Fibroblast Growth Factor 2, 10 ng/mL Epidermal Growth Factor, and 100 µM dibutyryl cAMP for twenty-five days to allow for differentiation. Cells were either used immediately for Figs. 1 and 2 or were treated for 24 h with 10 µM 27-OHC and 1 µM MG132 (Fig. 6). Cells were rinsed briefly with PBS, fixed in ice-cold acetone for 5 min, washed twice with PBS and incubated for 1 h with PBS containing 10% normal goat serum before applying PBS containing 5% normal goat serum and the following antibodies for the various figures: anti-TH mouse antibody (Cat. # MAB7566) (8 µg/mL R&D Systems, Minneapolis, MN, USA), anti-Neuron specific β-III Tubulin (Cat. # ab18207, RRID AB_444319) (Abcam, Cambridge, MA, USA), anti-α-synuclein rabbit antibody (Cat. # 2642S, RRID: AB_10695412) (1:500; Cell Signaling Danvers, MA, USA), anti-HSP70 antibody (Cat. # PA5-28003, RRID: AB_2545479) (1:1000; Thermo Fisher Scientific Waltham, MA USA), and anti-Dopamine Transporter (Cat. #MAB369, RRID: AB_2190413) (1:1000; EMD Millipore Temecula, CA USA) overnight at 4 °C. Cells were then washed three times with PBS (5 min each) and reacted to AlexaFluor 594 goat-anti-rabbit (Cat. # A11037, RRID AB_2534095) (Life Technologies, Carlsbad, CA, USA) and AlexaFluor 488 goat-anti-mouse antibody (Cat. # A11001, RRID AB_2534069) (Life Technologies, Carlsbad, CA, USA) in PBS containing 5% normal goat serum for 1 h at room temperature in the dark. Cells were washed three times with PBS for five minutes in the dark and mounted with Vectashield containing 4′,6-diamidino-2-pheylindole (DAPI) (Cat. # H-1500, RRID AB-2336788) (Vector Labs, Burlingame, CA USA), and visualized with a Leica DMI6000B microscope with a Leica DFC350 FX camera (Buffalo Grove, IL USA). Imaging was performed with a 10× (Fig. 1) and 20× (Figs. 2, 6) objective.

**Fig. 1:** Human dopaminergic neurons express Tyrosine Hydroxylase. Bright field microscopy of human dopaminergic neuronal precursor cells one day prior to the start of differentiation (**A**) and 25-day post differentiation (**B**). Immunofluorescence staining showing that the neurons express tyrosine hydroxylase, the rate limiting enzyme in dopamine synthesis (**C**; green) suggesting that these neurons are predominantly of dopaminergic origin. (**D**) is immunostaining with the neuron specific β-III Tubulin (red), and (**E**) is nuclear counterstain with DAPI (blue). **F** Overlay of tyrosine hydroxylase, neuron specific β-III Tubulin, and DAPI staining showing multiple neurons with nuclear and axonal/dendritic staining for tyrosine hydroxylase (arrows)

**Fig. 2:** Human dopaminergic neurons express Dopamine Transporter. A. Representative western blot (**A**) and optical density (**B**) of dopamine transporter (DAT) show the presence of DAT in the lysates from vehicle and 27-OHC-treated neurons. Immunofluorescence imaging shows immunopositive staining for DAT in untreated neurons (**C**; green). Immunofluorescence for the neuron specific β-III Tubulin marker (**D**; red) and for nuclear counterstaining with DAPI (**E**; blue). **F** Overlay of dopamine transporter, neuron specific β-III Tubulin, and DAPI showing both nuclear and cytoplasmic localization of DAT (arrows)

### Real time-rtPCR

Total RNA was extracted with the QuickGene RNA cultured cell HC kit S (Autogen, Holliston, MA). 1 µg of total RNA was reverse transcribed into cDNA with qScript cDNA SuperMix (Quanta Biosciences, Gaithersburg, MD). Real-time rtPCR was performed on the cDNA with taqman probes for the SNCA (Hs01103383_m1) gene (Applied Biosystems, Foster City, CA) and normalized to 18S rRNA. The data were quantified and expressed as fold-change compared to the control by using the ΔΔC_T_ method. Data are expressed as individual values with mean ± SEM and includes determinations made with (n = 3) and three technical replicates.

### Proteasome-glo™ caspase-like, chymotrypsin-like, and trypsin-like cell-based assays

Human primary dopaminergic neuronal precursor cells were grown in PriGrow IV medium containing 5% fetal bovine serum, 10 ng/mL Fibroblast Growth Factor 2, 10 ng/mL Glial-Derived Neurotrophic Factor, and 1% Penicillin–Streptomycin. Cells were maintained at 37 °C in a saturated humidity atmosphere containing 95% air and 5% CO_2_. Cells were cultured and passaged for 30 days prior to differentiation. Plates were coated with Poly l-Lysine and the cells were plated at a density of 10^4^ cells per cm^2^ with differentiation media consisting of PriGrow IV, 5% fetal bovine serum, 10 ng/mL Fibroblast Growth Factor 2, 10 ng/mL Epidermal Growth Factor, and 100 µM dibutyryl cAMP for twenty-five days to allow for differentiation. 96-well plates were then coated with Poly l-Lysine and differentiated cells were plated at a density of 10^3^ cells per well. Cells were treated in triplicate for 24 h with ethanol vehicle (control), 10 µM 27-OHC, and 1 µM MG132. Respective Proteasome-Glo™ substrates were added to cells for the three different types of proteasomal activity. The plates were placed on a plate shaker for 2 min at 700 rpm and incubated at room temperature for 15 min. The luminescence was measured using a luminometer and is expressed as Relative Luminescence Units (RLU) minus no cell media and reagent only blank wells. Data are expressed as individual values with mean ± SEM and includes determinations made in (n = 3).

### Statistical analysis

One-way analysis of variance (one-way ANOVA) was used to assess the significance of differences among the samples including more than two groups assuming the data was of parametric nature followed by Tukey’s post hoc test. Unpaired student’s t test was used to assess the significance of difference among the samples for the HSP70 western blots. Statistical analysis was performed with GraphPad Prism software 6.07. Quantitative data for western blotting analysis are presented as individual values with mean ± SEM with unit value assigned to control and the extent of differences among the samples being expressed relative to the unit value of control. Quantitative data for Real Time-rtPCR analysis are presented as individual values with mean ± SEM and expressed as fold-change from control.

## Results

### Human dopaminergic neurons express tyrosine hydroxylase and dopamine transporter

Human primary dopaminergic neuronal precursor cells were cultured and differentiated into human dopaminergic neurons according to the protocol provided by the vender. We acquired light microscopy images of pre (Fig. 1A) and post-differentiation (Fig. 1B). Twenty-five-day post differentiation, immunofluorescence imaging shows that the neurons express TH, the rate limiting enzyme in dopamine synthesis (Fig. 1C–F). We also performed western blotting to determine whether the cells express the dopamine transporter protein. Our results show that the differentiated neurons express dopamine transporter (DAT) and the DAT bands are present in absence or presence of the various concentrations of 27-OHC we used (Fig. 2A, B). There were no significant differences in the protein levels of DAT between the used concentrations of 27-OHC. Immunofluorescence assay corroborates the western blot results and shows that the untreated cells express DAT, (Fig. 2C, F).

### 27-OHC increases protein but not mRNA levels of α-synuclein

We determined the effects of increasing concentration of 27-OHC on the viability of dopaminergic neurons and found that there was no significant cell death with any of the chosen treatment concentrations (Fig. 3a). We then investigated the effects of 27-OHC on α-syn protein levels in human dopaminergic neurons. We found that 27-OHC significantly increases the levels of α-syn protein with 0.5 µM 27-OHC (*p* < 0.01), 1 µM 27-OHC (*p* < 0.001), and 10 µM 27-OHC (*p* < 0.001) (Fig. 3b, c). Real-time RT-PCR analysis demonstrates that 27-OHC does not affect the α-syn mRNA levels (Fig. 3d). This data suggests the mechanism by which 27-OHC increases α-syn protein levels in human dopaminergic neurons is through post-translational modifications or processing of the α-syn protein because 27-OHC does not appear to be modulating α-syn at a transcriptional level.

**Fig. 3:** 27-OHC does not kill cells and increases α-synuclein protein levels while mRNA levels remain unchanged. **a** Lactate Dehydrogenase assay shows that varying concentrations of 27-OHC do not elicit cell death relative to control untreated cells. Representative western blot (**b**) and optical density (**c**) of α-syn. Western blots are expressed as fold change over β-Actin. The amount of α-syn significantly increases with increased 27-OHC concentrations. **d** Real-time rt-PCR shows that 27-OHC does not increase *SNCA* mRNA. Data are expressed as individual values with mean ± SEM and includes determinations made in one experiment with (n = 3) and three technical replicates for LDH assay, two separate experiments with (n = 3) and three technical replicates for western blots, and one experiment with (n = 3) and three technical replicates for Real Time- rtPCR. **p < 0.01, ***p < 0.001 versus control

### The LXR agonist, GW3965, and the LXR antagonist, ECHS, do not affect α-synuclein mRNA or protein levels

We determined the extent to which 27-OHC increases α-syn through its cognate receptors LXRs as we have previously shown in human neuroblastoma SHSY5Y cells [21]. We utilized the LXR agonist GW3965 [37–39] and the LXR antagonist ECHS [21, 40] in these experiments. Figure 4a shows that 10 µM 27-OHC, 10 µM GW3965, 10 µM ECHS, and 10 µM 27-OHC + 10 µM ECHS did not kill the dopaminergic neurons relative to control as determined with the LDH assay. In order to test whether 27-OHC is activating LXRs in normal human dopaminergic neurons we performed western blots on ABCA1, a downstream protein of LXR activation. 27-OHC (*p* < 0.01) and GW3965 (*p* < 0.01) significantly increased the amount of ABCA1 protein while ECHS kept the levels near control. ECHS in combination with 27-OHC was not able to rescue ABCA1 levels back to baseline as this treatment also exhibited a significant increase in ABCA1 (*p* < 0.01) (Fig. 4b, c). These blots strongly suggest that 27-OHC is able to activate LXRs in normal human dopaminergic neurons. When probing for α-syn in western blotting we observed that only 27-OHC significantly increased α-syn protein levels while GW3965, ECHS, and 27-OHC + ECHS had no significant effect on α-syn protein content (Fig. 4d, e). To test the hypothesis that the effects of 27-OHC on α-syn are transcriptional through LXRs, we performed a real-time RT-PCR analysis in the presence of 27-OHC, GW3965, ECHS, and 27-OHC + ECHS and discovered that no treatments significantly affected α-syn mRNA content (Fig. 4f). This data strongly suggests that 27-OHC increases α-syn protein levels through a mechanism independent of transcriptional control by LXRs.

**Fig. 4:** The LXR agonist, GW3965, and the LXR antagonist, ECHS, do not affect α-synuclein protein or mRNA levels. **a** Lactate Dehydrogenase assay shows that 27-OHC, GW3965, ECHS, and 27-OHC + ECHS do not elicit significant cell death relative to control untreated cells. Representative western blot (**b**) and optical density (**c**) of ABCA1 expressed as fold change over β-Actin. 27-OHC and GW3965 both significantly increase the amount of ABCA1 protein levels. ECHS does not significantly alter the protein levels of ABCA1 while 27-OHC + ECHS significantly increases the amount of ABCA1. Representative western blot (**d**) and optical density (**e**) of α-syn. Western blots expressed as fold change over β-Actin. 27-OHC significantly increased the amount of α-syn protein levels while the LXR agonist GW3965 and LXR antagonist ECHS had no effects on α-syn protein levels. **f** Real-time rt-PCR shows that 27-OHC, GW3965, ECHS, and 27-OHC + ECHS do not significantly affect *SNCA* mRNA levels. Data are expressed as individual values with mean ± SEM and includes determinations made in one experiment with (n = 3) and three technical replicates for LDH assay, two separate experiments with (n = 3) and technical replicates for western blots, and one experiment with (n = 3) and three technical replicates for PCR. *p < 0.05, **p < 0.01, ***p < 0.001 versus control

### 27-OHC impairs proteasomal function and decreases HSP70 protein levels leading to increased α-syn protein levels

As the LXR transcriptional activity appears to not be involved in the 27-OHC-induced increase in α-syn protein levels we determined the potential role of 27-OHC in inhibiting the degradation of α-syn protein using ExPASy PeptideCutter, a tool that predicts potential cleavage sites cleaved by proteases in a given protein sequence. Our data shows that both 27-OHC and the proteasomal inhibitor MG132 reduce Caspase-like activity (Fig. 5a). The chymotrypsin-like and trypsin-like, the two proteasomal modes of α-syn degradation, are significantly inhibited by 27-OHC (Fig. 5b, c) as well as MG132. Our data demonstrates that MG132 and 27-OHC treatments both significantly increase α-syn protein levels versus vehicle-treated cells as shown with western blotting (Fig. 5d, e) and immunofluorescence imaging (Fig. 6A–L). This data strongly suggests that the 27-OHC-induced proteasomal inhibition plays a key role in the accumulation of α-syn protein. Our data also shows that 27-OHC significantly decreases while MG132 significantly increases HSP70 protein levels versus vehicle-treated cells as determined with western blotting (Fig. 5f, g). A significant decrease in HSP70 protein content could lead to abnormal cellular proteostasis as HSP70 is involved in protein folding and numerous degradation pathways, including the UPS, depending on which co-chaperones are involved. The significant decrease in HSP70 protein level caused by 27-OHC could possibly be the cause of proteasomal inhibition or another compromising event to cellular protein maintenance machinery involved in folding and degradation of proteins which is yet to be determined.

**Fig. 5:** 27-OHC inhibits proteasomal function and reduces HSP70 levels. 27-OHC and the proteasomal inhibitor MG132 significantly decrease Caspase-Like Proteasomal Activity (**a**), Chymotrypsin-Like Proteasomal Activity (**b**), and Trypsin-Like Proteasomal Activity (**c**). Representative western blot (**d**) and optical density (**e**) of α-syn. Western blots are expressed as fold change over β-Actin. 27-OHC and MG132 significantly increase the amount of α-syn protein. Representative western blot (**f**) and optical density (**g**) of HSP70 showing that while 27-OHC reduces HSP70 levels, treatment with MG132 dramatically increases HSP70 protein levels. Data are expressed as individual values with mean ± SEM and includes determinations made in one experiment with (n = 3) for the proteasomal assays and two separate experiments including (n = 3) and three technical replicates for the western blots. *p < 0.05, **p < 0.01, ***p < 0.001 versus control. ^†^*p* < 0.05, ^†††^*p* < 0.001 MG132 versus 27-OHC

**Fig. 6:** Both 27-OHC and the proteasomal inhibitor MG-132 increase α-syn protein levels. Immunofluorescene imaging shows that both 27-OHC (**E**) and MG132 (**I**) increase the immunostaining of α-syn compared to control untreated cells (**A**). Staining with the Neuron Specific βIII-Tubulin marker in control (**B**), 27-OHC-treated (**F**) and MG132-treated (**J**) neurons. Staining with the nuclear counterstain DAPI in control (**C**), 27-OHC-treated (**G**) and MG132-treated (**K**) neurons. The overlay shows multiple neurons exhibiting nuclear α-syn staining (arrows) in 27-OHC (**H**) and MG132 (**L**) treated neurons compared to untreated neurons (**D**)

## Discussion

Abnormal accumulation of α-syn protein is a characteristic of PD and other disorders collectively referred to as synucleinopathies. The causes of the accumulation of α-syn remain unknown, but genetic predisposition together with environmental factors are likely to contribute to the pathogenesis of synucleinopathies. 27-OHC is an active product of cholesterol metabolism made in the mitochondria of most cells by the enzyme CYP27A1 and serves many biological roles. This oxysterol has been shown to promote atherosclerosis via activation of proinflammatory processes [41], promotes breast and prostate cancers [42] and functions as a ligand of the LXRs [16]. LXRs, by means of gene transcription, regulate several metabolic pathways including lipid metabolism, glucose homeostasis, and inflammation [16]. We [21, 22] and other laboratories [29] have previously shown that the oxysterol 27-OHC evokes an increase in α-syn expression by mechanisms involving LXR activation in human neuroblastoma SHSY5Y cells. In this study, we determined the extent to which 27-OHC can regulate α-syn expression levels in human dopaminergic neurons, an in vitro model system that recapitulates synucleinopathies of PD type. We found that 27-OHC increases α-syn protein levels, activates LXR as shown by an increase in ABCA1, but fails to elicit a change in α-syn mRNA. GW3965, an LXR agonist and ECHS, an LXR antagonist also failed to elicit any change in α-syn protein or mRNA content suggesting there is no link between LXR and α-syn levels increase in the dopaminergic neuronal model. We took our investigation further to study proteasomal inhibition as a potential post-translational event that could contribute to the 27-OHC induced increase in α-syn protein levels. Proteasomes are large intracellular protein complexes whose main function is to degrade short-lived, damaged, and misfolded proteins by proteolysis. Proteasomes help control for the amount of proteins necessary for normal cellular functioning. In higher organisms, proteasomes are located both in the cytoplasm and nucleus. The most common form is the 26S proteasome, which contains one 20S core catalytic particle and normally one 19S regulatory particle at each side of the 20S core particle. The 20S core, which is concealed inside the 19S particles, is the active site of the proteasome which is responsible for its caspase-like, chymotrypsin-like, and trypsin-like activities. Initially, proteins targeted for degradation are tagged with several molecules of ubiquitin. Ubiquitin is covalently attached to target proteins by three sequential enzymatic steps: ubiquitin activation by E1 enzymes, ubiquitin conjugation by E2 enzymes, and ubiquitin ligation to target proteins by E3 enzymes. Ubiquitin is normally conjugated via its carboxy-terminal glycine to an internal lysine residue [43]. Following many rounds of ubiquitinylation a polyubiquitin chain is formed. This chain can function as a signal for degradation by the proteasome. The proteasome unfolds substrates and threads the polypeptide chains through the inner channel, where they are cleaved into short peptides [44]. After release from the proteasome, peptides are quickly processed into amino acids and recycled [45]. One approach to determine the functionality of the UPS is to assess the individual enzymatic activities involved in ubiquitin-dependent proteasomal degradation [46, 47]. Examining proteasomal function is the final stop of all ubiquitinylated proteins to be degraded and creates a bottleneck in the UPS pathway [47]. Therefore, it isn’t surprising that most studies focusing on the functionality of the UPS examine proteasomal function and not the individual enzymatic reactions leading up to it. However, this correlation of proteasomal activity and overall UPS impairment is complicated because it is presently unknown to what extent altered proteasomal activity affects the overall changes in degradation of ubiquitinylated proteins [47]. The ubiquitin proteasomal system (UPS) is a highly regulated system that controls the degradation of proteins involved in signal transduction, apoptosis, cell cycle progression and differentiation [48]. It is the chief pathway involved in the removal of damaged, misfolded and short-lived proteins within the cytoplasm and nucleus of cells. It functions by sequentially ubiquitinylating and degrading target proteins [47, 49, 50]. We show that 27-OHC increases α-syn protein levels through proteasomal inhibition in normal dopaminergic neurons that could potentially have implications in protein folding, UPS function and autophagy-lysosomal pathways of degradation. 27-OHC may potentially affect the UPS as this oxysterol has been shown to increase oxidative stress in astrocytes [51], and prolonged oxidative stress has been shown to decrease proteasomal function [52]. HSP70 uses its ATP hydrolysis-powered conformational changes to assist protein folding, disaggregation and degradation, and is a key contributor in cellular proteostasis. The decrease in HSP70 protein levels we observed could have numerous effects on cellular proteostasis. HSP70 is capable of being involved in various degradation pathways by the presence of specific chaperones and co-chaperones that aid in guiding the targeted protein to a specific degradation pathway (see [53] for a review). α-syn has been shown to bind HSP70 [54–56] and be degraded by the UPS and autophagy [32]. The extent to which a decrease in HSP70 affects proteasomal and/or autophagy is yet to be determined in future studies.

## Conclusions

In summary, we demonstrate that 27-OHC induces an increase in α-syn levels in human dopaminergic neurons. The mechanism involved in the α-syn increase does not appear to involve LXRs as we did not observe any significant changes in α-syn mRNA with 27-OHC or LXR agonist and antagonistic treatments. To the best of our knowledge, our results are the first to show that 27-OHC increases α-syn in dopaminergic neurons and that this increase may emanate from inhibition of the proteasomal function. Also, 27-OHC decreases levels of HSP70 protein which is involved in protein folding, and protein degradation through the UPS [53]. The extent to which a decrease in HSP70 protein levels leads to decreased protein folding and degradation through specific pathways needs to be further elucidated. All-together, our results potentially suggest that restoring proteasomal function and HSP70 protein levels may attenuate the 27-OHC-induced increase in α-syn protein levels in vitro and reduce α-syn accumulation that can increase the risk for synucleinopathies.

## Abbreviations

α-syn: α-synuclein
TH: tyrosine hydroxylase
27-OHC: 27-hydroxycholesterol
ECHS: 5a-6a-epoxycholesterol-3-sulfate
PD: Parkinson’s disease
LXR: liver X receptor
ABCA1: ATP-binding cassette transporter
HSP-70: heat shock protein 70
UPS: ubiquitin proteasomal system
